The article "Maximal Information Coefficient-Based Testing to Identify Epistasis in Case-Control Association Studies" was published in 2022. Journal: Comput Math Methods Med.

# Maximal Information Coefficient-Based Testing to Identify Epistasis in Case-Control Association Studies

**DOI:** 10.1155/2022/7843990

**Published:** 2022-02-15

**Authors:** Yingjie Guo, Zhian Yuan, Zhen Liang, Yang Wang, Yanpeng Wang, Lei Xu

**Affiliations:** ^1^School of Electronic and Communication Engineering, Shenzhen Polytechnic, 7098 Liuxian Street, Shenzhen 518000, China; ^2^Institute of Fundamental and Frontier Sciences, University of Electronic Science and Technology of China, No. 4 Block 2 North Jianshe Road, Chengdu 610054, China; ^3^Research Institute of Big Data Science and Industry, Shanxi University, 92 Wucheng Road, Taiyuan 030006, China; ^4^School of Life Science, Shanxi University, 92 Wucheng Road, Taiyuan 030006, China; ^5^Beidahuang Industry Group General Hospital, Harbin, China

## Abstract

Interactions between genetic variants (epistasis) are ubiquitous in the model system and can significantly affect evolutionary adaptation, genetic mapping, and precision medical efforts. In this paper, we proposed a method for epistasis detection, called EpiMIC (epistasis detection through a maximal information coefficient (MIC)). MIC is a promising bivariate dependence measure explicitly designed for rapidly exploring various function types equally and for interpreting and comparing them on the same scale. Most epistasis detection approaches make assumptions about the form of the association between genetic variants, resulting in limited statistical performance. Based on the notion that if two SNPs do not interact, their joint distribution in all samples and in only cases should not be substantially different. We developed a statistic that utilizes the difference of MIC as a signal of epistasis and combined it with a permutation resampling strategy to estimate the empirical distribution of our statistic. Results of simulation and real-world data set showed that EpiMIC outperformed previous approaches for identifying epistasis at varying degrees of heredity.

## 1. Introduction

Genome-wide association studies (GWAS) is an emerging research strategy for discovering associations between genetic variation (e.g., single nucleotide polymorphism (SNP)) and traits like human diseases. More than 71,000 SNPs have been confirmed to be related significantly to diseases [1–3] since the first GWAS study was published in *Science* in 2005 [4]. The majority of these markers, however, are common genetic variants with small effects. Even though the whole genome sequencing enables us to detect several rare variants with large effect, “missing heritability” for the complex disease remains extensive [5–7]. For instance, only 75% of the phenotypic variance of Alzheimer's disease has been explained by known variants [8]. One possible explanation for “missing heritability” is that complex diseases are polygenic, with multiple genes, environmental variables, and interactions involved in their etiology [9, 10]. Genetic interactions are thought to provide a potential answer to the problem of “missing heritability.” The solution may be partial, but it may help develop novel gene pathway topologies [11].

Epistasis is generally detected in two ways: biologically and statistically. Bateson and Mendel [12] introduced the concept of biological epistasis, which evaluates the interdependence of genetic variants. It occurs when the effect of one allele on one genetic mutation is dependent on the presence or absence of another genetic mutation and subsequently suppresses or activates the expression of other genes. Several studies reported novel epistasis in diseases. For instance, interactions between SNPs have been associated with pulmonary tuberculosis [13, 14], recurrent miscarriage [15], polycystic ovary syndrome [16], and many more [17–20]. These findings highlight the potential and significance of epistasis research.

Statistical epistasis, coined by Fisher [21], is defined as the deviation from additive effects of genetic mutations at separate loci in terms of their overall contribution to the model. Biological epistasis, on the other hand, refers to the physical interaction of two or more biological components. Studies in model organisms [22–24] have shown that epistasis found using computational and statistical approaches may be physiologically connected in these species. The presence of statistical epistasis, however, does not imply the presence of biological epistasis. Bridging the statistical and biological epistasis gap is a crucial step toward understanding the underlying genetic architecture of complex diseases.

Currently available approaches for detecting statistical epistasis can be divided into three groups depending on their strategy: exhaustive methods, search methods, and machine learning-based methods [25, 26]. Exhaustive methods have evaluated the association of all SNP combinations with phenotypes. Wan et al. [27] proposed BOOST, a multistage exhaustive approach that uses bitwise storage technology to speed up logistic regression test calculation. Zhang et al. [28] developed TEAM that calculates contingency tables by introducing a minimum spanning tree structure to detect pairwise SNP interactions. Ritchie et al. [29] used multifactor dimensionality reduction (MDR) to identify epistasis, which reduced the multiple SNP combinations into one dimension with high risk and low risk. It is one of the widely used methods in this field, and many methods have been developed based on it [30–33].

Exhaustive methods can effectively avoid omitting epistasis detection, but it requires massive computation. Stochastic techniques and heuristic searches are examples of search algorithms. The performance of stochastic methods involves random sampling and probability calculation. BEAM was created by Zhang and Liu [34] to find epistasis by partitioning SNPs into three nonoverlapping groups based on their posterior probability using Markov Chain Monte Carlo sampling. Schork et al. introduced EpiMODE [35], which combined the epistasis module idea with a Gibbs sampling strategy. Heuristic search is an approximation search guided by heuristic information that can reduce the search space and find the optimal solution effectively but may be limited by local optimal solutions. EpiACO [36] and AntEpiSeeker [37], both based on ant colony optimization, are examples of this sort of approach. Epi-GTBN [38] is an epistasis search approach that incorporates genetic algorithms to the Bayesian network heuristic search strategy.

SNP epistasis is also detected using machine learning-based approaches such as the neural network [39], support vector machine [40], random forest, or association rules [41]. SNPrule [42] is an epistasis detection method based on learning predictive rules, and by identifying the predictive rules involved in epistasis, higher-order epistasis may be inferred. EpiForest [43], random Jungle [44], and SNPInterforest [45] are examples of random forests that have been used in GWAS. They treated the random forest output as the most crucial variable set.

This paper introduces EpiMIC (epistasis detection via maximal information coefficient), an epistasis detection method that uses the maximal information coefficient (MIC) to identify marker-level interactions of complex diseases in case-control studies [14, 46]. MIC is a good bivariate dependency measure explicitly designed for rapid exploration of almost all types of data relationships, which means it can detect linear, exponential, and cyclical functions. Specifically, it can detect various function types equally, interpret them, and compare them on the same scale. We establish a statistic that utilizes the difference of MIC as an indicator of the occurrence of epistasis and also use the permutation resampling strategy to learn our statistic's empirical distribution. In simulated data sets with a variety of parameters, our method has demonstrated outstanding performance in finding underlying paired epistasis. Its use of WTCCC (Wellcome Trust Case Control Consortium) rheumatoid arthritis (RA) data shows accurate epistasis detection.

## 2. Materials and Methods

This section describes the EpiMIC statistical framework. The various parameter choices for simulation studies are presented to assess the power to detect type-I error and pairwise epistasis. Then, using the rheumatoid arthritis data set from the WTCCC database, we evaluated the efficiency of our method in a real-world setting.

### 2.1. EpiMIC

#### 2.1.1. Preliminaries and Notation

Suppose we have *n* random samples with a collection of *p* SNPs, then the observed genotypes *ℛ*^*p*^ can be represented by a *n* × *p* matrix:

(1) $$\begin{array}{c} G={\left[g_{l,i}\right]}_{l\in 1\cdots n,i\in 1\cdots p}, \end{array}$$

where *g*_*l*,*i*_ is the random variable that models the genotype for SNP *i* of *l*^th^ sample. It is a categorical variable with three levels denoted by *g*_*l*,*i*_ ∈ {*AA*, *Aa*, *aa*} = {0, 1, 2}. The homozygote genotypes are represented by *AA* and *aa*, whereas the heterozygote condition is represented by *Aa*. *A* and *a* denote the major and the minor alleles of SNP *i*, respectively. The value indicates the copy number of SNP *i*'s minor alleles. In case-control studies, *y*_*i*_ ∈ {0, 1} is a categorical label where 0 represents a control subject and 1 represents a case subject.

To determine whether there was a statistical interaction between two SNPs in a case-control study, we developed a statistic through the maximal information coefficient to quantify the strength of pairwise epistasis. We then used the permutation resampling strategy to estimate the statistic's empirical distribution. Intuitively, any pair of SNPs may have an original dependency or not without the phenotypic background. EpiMIC tried to capture the conditional dependency between a pair of SNPs under a disease status, which is the task-related correlation. It is based on the idea that because control samples are frequently picked at random, the epistasis pattern in case samples is more representative for understanding the underlying disease etiology. If there is no epistasis between two SNPs for disease, their dependence should show nothing significantly different in both cases and all samples; if they interacted under a disease, their dependency should be significantly different in cases and in all samples. Some methods can be used to calculate the dependency between two variables but may be limited by the functional form; for example, Pearson's correlation only measures linear dependence. Hence, we propose instead quantifying them using the maximal information coefficient.

#### 2.1.2. Maximal Information Coefficient

MIC [46] is an efficient measure of reliance for bivariate associations that encompasses a wide range of functional and not functional associations. It has two heuristic properties: generality and equitability. Generality means that if the sample size is sufficient, MIC covers not only certain types of functions but also various interesting associations or functional relationships that are not well modeled by a function, such as a superposition of functions. Equitability means MIC should assign identical ratings to similarly noisy associations of all kinds.

Let *D* ⊂ *ℛ*^2^ be a bivariate finite collection of ordered pairs, with *x* values and *y* values of *D* separated into *x* bins and *y* bins, respectively. An (*x*, *y*) grid is the term given to such a pair of partitions. The distribution *D*|_*G*_ for a grid *G* can be determined from the data points in *D* on the cells of *G*. It is calculated by taking the probability mass in each cell and dividing it by the proportion of data points in *D* that fall into that cell. Given a constant *D*, different grids *G* produce distinct distributions of *D*|_*G*_. With positive integers (*x*, *y*), define *I*^∗^(*D*, *x*, *y*) as

(2) $$\begin{array}{c} I^{*}\left(D,x,y\right)=\max I\left({\left.D\right|}_{G}\right), \end{array}$$

where the maximum is across all grids (*x*, *y*) and *I*(*D*|_*G*_) represents the mutual information of *D*|_*G*_.

The characteristic matrix *M*(*D*) of a bivariate data collection *D* is an infinite matrix with elements:

(3) $$\begin{array}{c} M{\left(D\right)}_{\left(x,y\right)}=\frac{I^{*}\left(D,x,y\right)}{\log\min\left\{x,y\right\}}. \end{array}$$

With Equation (3), the MIC of a bivariate data set *D* with *n* samples and a grid size smaller than *B*(*n*) is defined as follows:

(4) $$\begin{array}{c} \text{MIC}\left(D\right)=\underset{xy<B\left(n\right)}{\max}\left\{M{\left(D\right)}_{\left(x,y\right)}\right\}, \end{array}$$

where *ω*(1) < *B*(*n*) ≤ *O*(*n*^1−*ε*^) for some 0 < *ε* < 1. The function *B*(*n*) upper binds the sizes of the grids over which MIC searches. Usually, its default setting is *n*^0.6^ because it works well in practice.

To calculate *M*(*D*), it is optimized ideally on all possible grids. But in practice, MIC uses dynamic programming algorithms that optimize only a subset of possible grids for computational efficiency, and it seems to be approaching the true value of MIC.

MIC satisfies the following properties:

- Symmetry: MIC(*X*, *Y*) = MIC(*Y*, *X*)
- Comparability: MIC ∈ [0, 1], MIC = 0 denotes that two variables are independent statistically; MIC = 1 implies a strong association
- Generality: MIC could capture a wide range of relationships
- Equitability: MIC is robust to noisy relationships. It provides the same ratings to similarly noisy associations of various sorts

#### 2.1.3. Illustration of the EpiMIC Framework

Assume there are *n* samples in a case-control study, with *n*_2_ of them being cases. Let MIC_*n*_(*g*_*i*_, *g*_*j*_) be the sample correlation score between the *i*^th^ SNP and the *j*^th^ SNP. First, we calculated the MIC_*n*_^all^(*g*_*i*_, *g*_*j*_) for all the samples and MIC_*n*_2__^*D*^(*g*_*i*_, *g*_*j*_) for case samples. Second, we devised a statistic ∆MIC = |MIC_*n*_^all^(*g*_*i*_, *g*_*j*_) − MIC_*n*_2__^*D*^(*g*_*i*_, *g*_*j*_)|/MIC_*n*_^all^(*g*_*i*_, *g*_*j*_) to compare the MIC in cases and in all samples. ∆MIC denotes how dissimilar the relationship (*g*_*i*_, *g*_*j*_) was in cases and across all samples. The greater the ∆MIC, the more likely it is that *g*_*i*_ and *g*_*j*_ interacted.

We wanted to learn the empirical distribution of ∆MIC^0^ under the null hypothesis to derive a *p* value. In this case, we employed a nonparametric permutation strategy: first, shuffled the *y* with *m* times, computed ∆MIC by the same procedure described above, and used the resultant sample distribution as an estimate for the distribution of ∆MIC. If the outcome of these *m* permutations is ∆MIC^1^, ⋯, ∆MIC^*m*^, an estimated *p* value under the null hypothesis is

(5) $$\begin{array}{c} p=\frac{\left|\left\{i:∆\text{MI}{\text{C}}^{i}\geq ∆\text{MI}{\text{C}}^{0}\right\}\right|}{m}. \end{array}$$

In Algorithm 1, we summarized the EpiMIC procedure and showed the whole workflow in Figure 1.

### 2.2. Simulation Study

To evaluate EpiMIC's ability to control type-I error and detect marker-based pairwise epistasis, we compared EpiMIC with BEAM [34], MDR [29], BOOST [27], and Epi-GTBN [38].

#### 2.2.1. Simulation with GAMETES

The performance of the EpiMIC to detect marker-based, pairwise epistasis was examined in this simulation study. We assigned 10 SNPs to each simulation data set. There were two functional SNPs and eight nonfunctional SNPs among them. To produce the simulated genotype data, we used the freely accessible program GAMETES [47]. This program was created to produce pure and strict epistasis models, which are the most challenging to discover if all *n*-loci are included in the disease model. Because of this requirement, these models are a desirable gold standard for simulation research on complex epistasis [47, 48].

*(1) Type-I Error Evaluation*. Type-I error demonstrates a method's capacity to reject the null hypothesis when it is true. We utilized the GAMETES to create two custom disease models without epistasis (Table 1). The baseline odd was denoted by *γ*. We conducted the simulation for each model 100 times with the following sample size *n* ∈ {1*k*, 2*k*, 3*k*, 4*k*, 5*k*}, *γ* = 1, and *θ* = 5. The threshold of significance was fixed at 0.05.

*(2) Evaluation of Test Power*. The power of a test reflects the likelihood that the procedure will properly accept the alternative hypothesis when the null hypothesis is false. This simulation study used two experimental setups: epistasis models without marginal effects (NME) and epistasis models with marginal effects (ME).

For each parameter setting in the NME scenario, we created 100 data sets. The power under each parameter value was stated as the frequency at which the approach successfully rejects the null hypothesis at a significance level of *α* = 0.05.

- We used *h* ∈ {0.005, 0.01,0.025,0.05,0.1,0.2} and two distinct minor allele frequencies (MAF) ∈ {0.2,0.4} to analyze the influence of heritability *h*. Five models were developed for each parameter combination, yielding 60 models following Hardy-Weinberg proportions. For all these models, population prevalence was set to 0.2, and the sample size was set to 4,000. The five models were labeled M1 to M5, and they were sorted in general by rising customized odds ratio (COR) using GAMETES. COR is a detectability statistic derived directly from the genetic model. The higher the value, the simpler it is to identify epistasis
- To assess the effect of sample size, we set heritability to 0.025, MAF ∈ {0.2, 0.4}, and prevalence to 0.2, with a sample size of 10,000. Then, using this big data set, 100 data sets were created at random for each of the sample size *n* ∈ {1*k*, 2*k*, 3*k*, 4*k*, 5*k*}. In this case, we had a total of 1,000 data sets

In the ME scenario, we generated six models in accordance with Namkung et al. [49]. For each model, 100 replicated data sets with balanced case subjects and control subjects were constructed with a sample size of 4,000 (Table 2).

For BEAM, MDR, BOOST, and Epi-GTBN, let the number of data sets where they identified the epistasis correctly be *m*_1_, then the power can be determined using the following formula:

(6) $$\begin{array}{c} \text{power}=\frac{m_{1}}{100}. \end{array}$$

We ran BEAM and Epi-GTBN with the default parameter setting. MDR and BOOST had no parameters to be specific. In EpiMIC, *n*^0.7^ ~ *n*^0.8^ is effective experimentally. We use *n*^0.8^ as a default parameter.

### 2.3. Experiments Using Data from Rheumatoid Arthritis

To test EpiMIC's capacity to handle true epistasis in a case-control data set, we examined the susceptibility of a series of pairings of SNPs in rheumatoid arthritis (RA), an inflammatory disease characterized by pannus development in synovial joints and cartilage and bone loss. The detailed data set construction can be found in our previous work [48].

## 3. Results and Discussion

All results were obtained on a workstation equipped with an Intel Xeon CPU E5-2620 v2 @ 2.10 GHz, 96 GB of DDR3, R 4.0.3, and RStudio programming implementation.

### 3.1. Simulation Study

#### 3.1.1. Type-I Error Evaluation

For type-I error, we set MAF to 0.2 and population prevalence to 0.2, then ranged sample sizes from 1,000 to 5,000. For the no-effect model without epistasis, all the methods tested had a type-I error comparable to the significance level *α* = 0.05 (Table 3(a)). For the disease model without epistasis, but with one marginal SNP, BEAM and BOOST still controlled type-I error, although MDR, Epi-GTBN, and EpiMIC had little inflation. The result implied that we should choose a lower significance level in practical application to reduce the probability of false positive results.

#### 3.1.2. Evaluation of the Power of EpiMIC

*(1) The Influence of Heritability*. We investigated two types of epistasis disease models to assess the statistical strength of our EpiMIC and the other four methods: epistasis models without marginal effects (NME) and epistasis models with marginal effects (ME).

In the NME scenario, we examined 12 heritability-MAF combinations, with heritability ranging from 0.005 to 0.2 (Table 4). Table 4's bold font indicates the best-performing approach in each model for a given heritability-MAF combination. It is worth noting that a higher value suggests better performance. Except for the disease model *M*1 with *h* = 0.005 with MAF = 0.2, EpiMic was slightly better than other methods. For most parameter combinations, EpiMic had the same great performance as BOOST and Epi-GTBN. The statistical power of all the methods achieved 1 when MAF = 0.2, *h* > 0.01 and MAF = 0.4, *h* > 0.005 except for BEAM.

Heritability had a significant impact on the power of all methods, and the power increased monotonically with an increase in *h* under a certain MAF (Table 5). Heritability ranged from 0.005 to 0.01, and all methods demonstrated a consistent rising trend (Table 5). The power was also affected by the epistasis SNP pair's minor allele frequencies (MAF). Although BEAM fluctuated under model M1 with MAF = 0.4 and *h* = 0.05, for other methods, the increase in MAF was evident in the improved performance, especially when *h* = 0.005. Heritability is the effect size of epistasis. When it was small, the larger MAF increased the chances for causal genotypic combinations of epistasis SNP pairs to emerge in simulation data sets. For example, for the cases of *h* = 0.005, the average power of BEAM was 0.876 with MAF = 0.2, which was lower than 0.912 for MAF = 0.4. Although the performance of the methods under the same model was different, the epistasis detected by the high-power method did not entirely cover epistasis detected by the low-power method. Because these methods were based on different definitions of epistasis, the methods could not simply replace each other; instead, they had a complementary relationship.

It is worth mentioning that, as compared to BEAM or MDR, EpiMIC, BOOST, and Epi-GTBN were more stable for disease models M1 to M5 with varying COR under the same heritability-MAF combination. In the ME scenario, the power to detect epistasis for all methods achieved a 1 that the epistasis disease model with marginal effect was easier to analyze than models without marginal effect.

*(2) The Influence of Sample Size*. Let the sample size be *n* ∈ {1*k*, 2*k*, 3*k*, 4*k*, 5*k*}, with *h* = 0.005, and MAF = 0.2 (Figure 2). As the sample size increased, the power of all methods increased almost monotonically. A larger sample size corresponds to improved performance in all methods.

In conclusion, EpiMIC had superior or comparable performance to detect purely and strictly epistasis in simulation studies, which was the most difficult disease-related patterns with or without marginal effects. EpiMIC benefited from the powerful ability of MIC to capture a wide range of relationships and our designed statistic ∆MIC. If two SNPs interacted under a specific disease model, SNPs showed a more obvious relationship in some cases. Adding control samples decreases the strength of this relationship.

However, the nature of EpiMIC made it likely that it was affected by linkage disequilibrium (LD); because LD is a strong dependency, SNPs in a strong LD block may produce false positives.

### 3.2. Experiments Using Rheumatoid Arthritis Data

RA is an autoimmune disease in which IL-6, RANK, and TNF − *α* are key hereditary risk factors [50]. In the RA investigation, each unique SNP pair of the hsa05323 pathway was analyzed, yielding *C*_385_^2^ = 73, 920 total pairings for 385 SNPs. We chose 522 results with a significance level *α* = 0.005; after filtering SNP pairs in the same gene, we got 517 epistasis to do the following analysis.

We generated the epistasis network (Figure 3) from 517 epistasis using the network analysis software Gephi, in which the nodes were the SNPs with epistasis and the edge indicated the epistasis relationship. We generated Figure 3 by running the Multigravity Force Atlas algorithm, which prevented nodes from overlapping and controlled the scale of the expansion of the graph while clustering interconnected nodes. The degree of each node represents the number of epistasis that it was involved in, and the edge was weighted by the MIC of pairs of SNPs in case samples. The average degree of the network was 3.009. We filtered the nodes with degree < 5, then ordered the node size and color by its degree. Nodes labeled purple were the top 15 nodes ranked by the node's degree.

Table 6 gives a detailed information of the top 15 nodes, which included their degree, the gene where the SNP was located, and the genes where the interacting SNPs were located. We grouped the interacting SNPs into genes. The higher the node's degree was, the greater the chance that it interacted with more genes. But the number of genes that showed epistasis did not increase monotonically with the degree of a node; due to the different numbers of SNPs that were contained in each gene in the data set and their underlying interval LD pattern, one SNP may be detected as epistatic with multiple SNPs in the LD region from a long gene. From the network, we found some valuable hub genes, such as IL15, CD28, Ang1, Tie2, LFA1, and TLR4, which had at least five interacting genes in the RA pathway. For instance, IL-15 [51], which is a member of the 4 *α*-helix bundle cytokine family, was detected in the serum of RA patients and synovial fluid and in mouse models of arthritis. In addition, the administration of IL-15 led to the development of severe inflammatory arthritis, indicating that IL-15 may be related to RA treatment. Targeting IL-15 is very critical and valuable.

We also analyzed the top 10 epistasis ranked by the MIC in case samples for each pair of SNPs (Table 7) and found that five of the top 10 results were supported by prior research [52–55]. For example, the first epistasis was between gene CD80 (rs4675363) and CTLA4 (rs1427676). Costimulatory molecules have a crucial role in the immunoregulatory regulation of T lymphocyte-mediated immunological and inflammatory responses [53]. The best-studied costimulatory signaling pathway was CD28/CTLA4-CD80/CD86. CTLA-4 is a structural homolog of CD28, and it binds the CD80 and CD86 ligands. CTLA-4, on the other hand, has a 20-to-50-fold greater affinity to CD28, which gives a different regulatory function for CTLA to downregulate T cell immunity while allowing CD28 to initiate amplification and to maintain the positive immunity of T cells. T cells were not stimulated abnormally due to the tight and coordinated costimulation signaling pathway of CD28/CTLA4-CD80/CD86.

## 4. Conclusions

Epistasis between genetic variants is ubiquitous and crucial in uncovering the underlying genetic structure of complex diseases and traits. In this paper, we developed EpiMIC (epistasis detection via maximal information coefficient), which combined maximal information coefficient (MIC) with permutation strategy for case-control studies in GWAS. We transformed the epistasis detection problem by measuring the degree of difference of MIC between pairwise SNPs in cases and in all samples. The method benefits from the powerful ability of MIC to explore various function types equally and to interpret and compare them on the same scale. Because of the weak assumptions about the nature of epistasis and MIC's powerful and practical capacity to capture complicated functional and nonfunctional correlations, our method accurately and effectively recognized additional sorts of interpretable epistasis.

To assess EpiMIC's performance, we conducted simulated and retrospective investigations. For most of the settings tested, EpiMIC's statistical power to detect epistasis was better or equivalent to prior methods, and its power grew monotonically with heritability, MAF, and sample size. Based on a test of type-I error, the method was shown to be stable to sample size. Simulation results also indicated that epistasis detected by the high-power method did not entirely cover epistasis detected by the low-power method. These methods were based on different definitions of epistasis that methods could not simply replace each other but had a complementary relationship. In our analysis of real data, we found several key genes of RA from an epistasis network and significant epistasis that was supported by prior research. We found that local LD inflated EpiMIC's statistical power slightly. SNP pairs in the same gene with a LD pattern were detected as epistasis occasionally. In practice, we suggest filtering out SNP pairs within a local LD structure or select tagSNPs to detect epistasis. Moreover, due to different sequencing coverage, some causal SNPs may be missing in some data sets, and only markers linked to it are found to be epistasis. Therefore, it would be better to locate the interacting genes through marker-based epistasis first and then to combine more biological information to locate the real causal epistasis. In conclusion, EpiMIC is a useful addition to the current toolkit of statistical methods for elucidating epistasis in GWAS case-control studies.

## Figures and Tables

**Figure 1:** Illustration of the EpiMIC framework for pairwise epistasis detection.

**Figure 2:** The statistical power of simulation studies for BEAM (blue), BOOST (orange), MDR (green), Epi-GTBN (red), and EpiMIC (purple) under disease model with heritability = 0.005, MAF = 0.2, population prevalence = 0.2, and sample sizes that ranged from 1,000 to 5,000.

**Figure 3:** Variant network of rheumatoid arthritis results from the EpiMIC model with identified SNP pairs. The nodes were SNPs, and the edges represented the epistasis relationship. Node size and color reflected the number of epistasis that the node involved in. Edge thickness indicated the maximal information coefficient of SNPs in case samples. The node labels with highlights were the top 15 SNPs ranked by node degree.

**Algorithm 1:** EpiMIC.

**Table:** (a) No effect model

	AA	Aa	aa
BB	*γ*	*γ*	*γ*
Bb	*γ*	*γ*	*γ*
bb	*γ*	*γ*	*γ*

**Table:** (b) One marginal recessive model

	AA	Aa	aa
BB	*γ*	*γ*	*γ*
Bb	*γ*	*γ*	*γ*
bb	*γ*(1 + *θ*)	*γ*(1 + *θ*)	*γ*(1 + *θ*)

**Table 2:** The detailed information of the six disease models with marginal effects, which included prevalence, MAF, and penetrance for each combination of genotypes.

Models	Prevalence	MAF	Genotypes								
			AABB	AABb	AAbb	AaBB	AaBb	Aabb	aaBB	aaBb	aabb
Model 1	0.050	0.1	0.061	0.017	0.017	0.017	0.136	0.136	0.017	0.136	0.136
Model 2	0.050	0.1	0.060	0.021	0.021	0.021	0.116	0.116	0.021	0.116	0.116
Model 3	0.046	0.1	0.030	0.080	0.090	0.090	0.010	0.010	0.070	0.040	0.000
Model 4	0.026	0.1	0.030	0.010	0.020	0.010	0.090	0.050	0.020	0.050	0.070
Model 5	0.017	0.1	0.020	0.005	0.020	0.007	0.070	0.001	0.003	0.080	0.090
Model 6	0.052	0.2	0.044	0.066	0.073	0.069	0.021	0.007	0.042	0.073	0.054

**Table:** (a) No effect disease model

Methods	Sample size			
	1,000	2,000	3,000	4,000	5,000
BEAM	0	0	0	0	0
BOOST	0	0	0	0	0
MDR	0.03	0.02	0	0.01	0.04
Epi-GTBN	0.01	0	0.02	0.01	0.05
EpiMIC	0.02	0.03	0.05	0.02	0.04

**Table:** (b) Marginal disease model

Methods	Sample size			
	1,000	2,000	3,000	4,000	5,000
BEAM	0	0	0	0	0
BOOST	0	0	0	0	0
MDR	0.04	0.06	0.06	0.08	0.06
Epi-GTBN	0.06	0.07	0.06	0.08	0.11
EpiMIC	0.03	0.03	0.06	0.05	0.03

**Table 4:** The statistical power of simulation studies for BEAM, BOOST, MDR, Epi-GTBN, and EpiMIC with *h* ∈ {0.005, 0.01, 0.025, 0.05, 0.1, 0.2} and MAF ∈ {0.2, 0.4}. There are five models for each heritability-MAF combinations. The best-performing approach for each model is shown with a bold font. The results of some heritability-MAF combinations are not listed in the table because all methods under these parameter combinations are 1. These parameter combinations include MAF = 0.2 with *h* ∈ {0.025, 0.05, 0.1, 0.2} and MAF = 0.4 with *h* ∈ {0.01, 0.025, 0.2}.

MAF	Heritability	Method	Models				
			M1	M2	M3	M4	M5
0.2	0.005	BEAM	0.53	0.95	0.95	0.98	0.97
		BOOST	0.96	**1**	**1**	**1**	**1**
		MDR	0.14	0.84	**1**	**1**	**1**
		Epi-GTBN	0.94	**1**	**1**	**1**	**1**
		EpiMIC	**0.98**	**1**	**1**	**1**	**1**
	0.01	BEAM	1	1	1	1	1
		BOOST	1	1	1	1	1
		MDR	0.34	0.99	1	1	1
		Epi-GTBN	1	1	1	1	1
		EpiMIC	1	1	1	1	1

0.4	0.005	BEAM	0.87	0.93	0.9	0.93	0.93
		BOOST	**1**	**1**	**1**	**1**	**1**
		MDR	0.99	**1**	**1**	**1**	**1**
		Epi-GTBN	**1**	**1**	**1**	**1**	**1**
		EpiMIC	**1**	**1**	**1**	**1**	**1**
	0.05	BEAM	0.76	1	1	0.98	1
		BOOST	1	1	1	1	1
		MDR	1	1	1	1	1
		Epi-GTBN	1	1	1	1	1
		EpiMIC	1	1	1	1	1

**Table 5:** Average power for the methods BEAM, BOOST, MDR, Epi-GTBN, and EpiMIC to detect epistasis under 12 heritability-MAF combinations.

MAF	Heritability	Methods				
		BEAM	BOOST	MDR	Epi-GTBN	EpiMIC
0.2	0.005	0.876	0.992	0.796	0.988	0.998
	0.01	1	1	0.866	1	1
	0.025	1	1	1	1	1
	0.05	1	1	1	1	1
	0.1	1	1	1	1	1
	0.2	1	1	1	1	1

0.4	0.005	0.912	1	0.998	1	1
	0.01	1	1	1	1	1
	0.025	1	1	1	1	1
	0.05	0.948	1	1	1	1
	0.1	1	1	1	1	1
	0.2	1	1	1	1	1

**Table 6:** Detailed information of the top 15 nodes ranked by the node's degree of SNP epistasis network generated using EpiMIC with RA data. The column “corresponding gene” indicates the gene where SNP was located, and the column “gene interaction” shows the genes where the interacting SNPs were located.

rsID	Corresponding gene	Degree	Gene interaction
rs10805069	IL15	12	GM-CSF, Tie2, TLR4, MMP3, FLT1
rs4796119	CCL2	11	M-CSF, CD28, CTLA4, Ang1
rs684	LFA1	10	M-CSF, Ang1, CTSL, RANK, LFA1
rs10490573	CD28	9	CD80, IL15, Ang1, Tie2, CCL2, CCL5, LFA1
rs10505107	Ang1	9	TGF*β*, CXCL1, IL15, TLR4, MMP3
rs11938228	CXCL1	9	IL1, IL6, Ang1, APRIL
rs3850890	CD80	9	TLR2, MMP3, IFN*γ*, AP1, CD28
rs1283659	Ang1	9	CD28, CXCL1, FLT1, CCL2
rs534129	Tie2	9	IL15, Ang1,TLR4, MMP1, MMP3
rs10519613	IL15	8	IL1, IL6, Ang1, APRIL
rs7855140	TLR4	8	IL15, IL17, Tie2, MMP1, IL18
rs544354	IL18	8	IL15, Tie2
rs6808536	CD80	8	M-CSF, Tie2, MMP3, FLT1
rs17069845	RANK	8	TLR2, Tie2
rs2367291	IL15	8	IL8, Tie2, FLT1, RANK, LFA1

**Table 7:** Detailed information of the top 10 epistasis ranked by the MIC in case samples for each pair of SNPs and genes where SNPs were located. The column “Ref” references the literature that showed the regulatory relationship between two genes.

rsID of SNP1	rsID of SNP2	Corresponding gene 1	Corresponding gene 2	Ref
rs4675363	rs1427676	CD28	CTLA4	[52]
rs7537752	rs6574222	M-CSF	FOS	[53]
rs4422395	rs7037246	TLR2	TLR4	
rs13285984	rs1634507	Tie2	CCL4	
rs12089727	rs6808536	MCSF	CD80	
rs2564594	rs1800795	TLR2	IL6	[54]
rs246841	rs266089	GM-CSF	CXCL12	[51]
rs550982	rs1569328	Tie2	AP1	
rs951759	rs266089	Ang1	CXCL12	
rs2256849	rs1474552	FLT1	ITGB2	

## Data Availability

Publicly available data sets were analyzed in this study. This data can be found here: https://www.wtccc.org.uk/info/access_to_data_samples.html.
